The article "Neuroprotective effects of the immunomodulatory drug FK506 in a model of HIV1-gp120 neurotoxicity" was retracted in 2026. Reasons: duplicated images; overlap with earlier publications; unreliable data; concerns about the data.

# Neuroprotective effects of the immunomodulatory drug FK506 in a model of HIV1-gp120 neurotoxicity

**DOI:** 10.1186/s12974-016-0585-8

**Published:** 2016-05-24

**Authors:** Jerel A. Fields, Cassia Overk, Anthony Adame, Jazmin Florio, Michael Mante, Andrea Pineda, Paula Desplats, Edward Rockenstein, Cristian Achim, Eliezer Masliah

**Affiliations:** Department of Pathology, University of California San Diego, La Jolla, CA USA; Department of Neurosciences, University of California San Diego, La Jolla, CA USA; Department of Psychiatry, University of California San Diego, La Jolla, CA USA

**Keywords:** FK506, gp120, HIV, Neuro-inflammation

## Abstract

**Background:**

HIV-associated neurocognitive disorders (HAND) continue to be a common morbidity associated with chronic HIV infection. It has been shown that HIV proteins (e.g., gp120) released from infected microglial/macrophage cells can cause neuronal damage by triggering inflammation and oxidative stress, activating aberrant kinase pathways, and by disrupting mitochondrial function and biogenesis. Previous studies have shown that FK506, an immunophilin ligand that modulates inflammation and mitochondrial function and inhibits calcineurin, is capable of rescuing the neurodegenerative pathology in models of Parkinson’s disease, Alzheimer’s disease, and Huntington’s disease. In this context, the main objective of this study was to evaluate if FK506 could rescue the neuronal degeneration and mitochondrial alterations in a transgenic (tg) animal model of HIV1-gp120 neurotoxicity.

**Methods:**

GFAP-gp120 tg mice were treated with FK506 and analyzed for neuropathology, behavior, mitochondrial markers, and calcium flux by two-photon microscopy.

**Results:**

We found that FK506 reduced the neuronal cell loss and neuro-inflammation in the gp120 tg mice. Moreover, while vehicle-treated gp120 tg mice displayed damaged mitochondria and increased neuro-inflammatory markers, FK506 rescued the morphological mitochondrial alterations and neuro-inflammation while increasing levels of optic atrophy 1 and mitofusin 1. By two-photon microscopy, calcium levels were not affected in the gp120 tg mice and no effects of FK506 were detected. However, at a functional level, FK506 ameliorated the gp120 tg mice hyperactivity in the open field.

**Conclusions:**

Together, these results suggest that FK506 might be potentially neuroprotective in patients with HAND by mitigating inflammation and mitochondrial alterations.

## Background

In recent years, highly effective combined antiretroviral therapies (cART) have had remarkable success in reducing the morbidity and mortality among patients with HIV [1]; however, HIV-associated neurocognitive disorders (HAND) continue to be a significant problem [2, 3]. HIV enters the CNS in macrophages and T cells early in the progression of the disease causing neuro-inflammatory and neurodegenerative pathology [4], a condition prevalent in the pre-cART era known as HIV encephalitis (HIVE). The effectiveness of the cARTs has shifted HIVE from a subacute condition to a low-level chronic disorder that is often associated with mild neurodegenerative pathology and mild HAND [5, 6].

HIV-1 proteins released from infected cells can lead to neurodegeneration in patients with HAND through a variety of mechanisms [7, 8]. For example, HIV-1 proteins such as gp120, Tat, and Nef activate apoptotic pathways [9], dysregulate calcium homeostasis [10, 11], and promote excitotoxicity [12, 13] and oxidative stress [14, 15]. In the CNS, secreted HIV-1 proteins have also been shown to alter autophagy pathways [16–18], aberrantly activate kinases, and hyperphosphorylate microtubule-associated protein tau [19, 20]. In addition, recent studies have shown that secreted HIV-1 proteins can lead to neurodegeneration by interfering with mitochondrial bioenergetics [21] and biogenesis [21, 22], which is similar to alterations in mitochondrial biogenesis that have been reported in patients with Parkinson’s disease (PD) [23], Alzheimer’s disease (AD) [24], and Huntington’s disease (HD) [25].

Mitochondrial biogenesis is partially regulated through mitochondrial fusion and fission events [26]. Fission is dependent upon the GTPase dynamin-related protein, (DRP) 1, and appears to be crucial for regulating mitophagy, as well as general mitochondrial distribution allowing mitochondria-organelle-contacts, Ca+ regulation, and ATP supply to distant regions such as axonal and dendritic synapses in neurons [27–29]. Fusion may serve as a stress response to protect cells from apoptotic cell death [30] and mitophagy [31]. Mitochondrial fusion is dependent on mitofusin (MFN) 1 and 2 and optic atrophy 1 (OPA1), and an imbalance of fusion and/or fission protein activity may lead to dysfunction and cell death [32].

Alterations in mitochondrial fusion/fission have been proposed to play an important role in neurodegenerative disorders [33, 34]. We have recently reported that in the brains of patients with HAND and in gp120 transgenic (tg) mice levels of MFN1, OPA1, a mitochondrial dynamin-like 120 kDa protein, and DRP1 were altered [21]. These changes are accompanied by enlarged mitochondria and alterations in mitochondrial bioenergetics [21]. Previous studies have shown that FK506, an immunophilin ligand [35, 36] that modulates mitochondrial function [37] and inhibits calcineurin and p38 mitogen-activated protein kinase (MAPK) activity [38–40], is capable of rescuing the neurodegenerative pathology in models of AD [41], PD [42] and HD [25]. In this context, the main objective of this study was to evaluate if FK506 would rescue the neuronal degeneration and mitochondrial alterations in a transgenic animal model of HIV-1 gp120 neurotoxicity. For this purpose, GFAP-gp120 tg mice were treated with FK506 and analyzed for neuropathology, calcium function, and behavior. We found that FK506 is neuroprotective in the gp120 tg model and ameliorates mitochondrial alterations and neuro-inflammation. These results suggest that FK506- or FK506-like analogues might be potentially useful managing the neurobehavioral alterations in patients HAND.

## Methods

### Generation of gp120 tg mice and treatments

For these studies, we utilized an animal model of HIV-1-protein-mediated neurotoxicity, which expresses high levels of gp120 under the control of the glial fibrillary acidic protein (GFAP) promoter [43]. These mice develop neurodegeneration accompanied by astrogliosis, microgliosis, and behavioral deficits [43]. As previously described [44], 12-month old non-tg and gp120 tg animals (total of 40 mice; *n* = 10 per group) received daily intraperitoneal (IP) injections with saline (vehicle) alone or FK506 (VWR International, Brisbane, CA) at a concentration of 5 mg/kg for 4 weeks. The mice were sacrificed following behavioral testing, and brains were removed for biochemical analyses of frozen or immunocytochemical analyses of fixed brain tissues. UCSD is an Institutional Animal Care and Use Committee accredited institution and the Animal Subjects Committee approved the experimental protocol (UCSD IACUC Protocol S02221) followed in all studies according to the Association for Assessment and Accreditation of Laboratory Animal Care International guidelines.

### Behavioral testing in the open field

The open-field locomotor test was used to determine basal activity levels of study subjects (total move time) during a 15-min session. Spontaneous activity in an open field (25.5 × 25.5 cm) was monitored for 15 min using an automated system (Truscan system for mice; Coulbourn Instruments, Allentown, PA). Animals were tested within the first 2–4 h of the dark cycle after being habituated to the testing room for 15 min. The open field was illuminated with an anglepoise lamp equipped with a 25-W red bulb. Animals were tested at 12 months of age (after 4 weeks of treatment). Time spent in-motion was automatically collected 3 × 5 min time bins using the TruScan software. Data were analyzed for both the entire 15-min session and for each of the 5-min time blocks.

### Two-photon microscopy and calcium imaging

A separate subset of non-tg and gp120 tg mice (total = 16, *n* = 4 per group, 12 m/o) was anesthetized with isoflurane (3 % initially, followed by 1–2 % during surgical procedures (tracheotomy, cannulation of femoral artery, and cortical exposure)). Surgical procedures were performed as previously described [42, 45]. During data acquisition, anesthesia was maintained with *α*-chloralose (50 mg kg^−1^) and pancuronium (0.4 mg/kg). Mice were ventilated with 30 % O_2_ in air (~100 bpm). Expired CO_2_ (CI240, Columbus instruments), heart rate, blood pressure (BP1, World Precision Instruments), and body temperature (Homeothermic blanket, Harvard Apparatus) were monitored continuously. Blood gas (Rapidlab 248, Siemens) was measured at the start of data acquisition to adjust the respiration parameters to achieve pCO_2_ 35–45 mmHg, pO_2_ 100–180 mmHg, and pH 7.35–7.45. A group of gp120 mice (*N* = 4) were treated with FK506 (5 mg/kg dissolved in 10 % ethanol 90 % saline, intra-arterial) 1 h before imaging. The calcium indicator Oregon Green 488 BAPTA-1AM (OGB, green) was loaded by microinjection [46], and glial marker sulforhodamine 101 (SR101, red) was applied topically to the brain. Images were obtained using an Ultima two-photon laser scanning microscopy system from Prairie Technologies, equipped with an Ultra II femtosecond laser (Coherent) tuned to 800 nm. A single electrical stimulus (100 μs, 1 mA) was delivered to the contralateral whisker pad. Within each ~50 × 100 μm field of view (FOV), neuronal cell bodies were imaged in a frame scan mode with a target acquisition rate of 10 Hz. Fifteen stimulus trials with interstimulus intervals (ISI) of 15 s were presented for each FOV and for each of the two stimulus conditions.

For the extraction of time courses, masks corresponding to individual neuronal bodies were segmented from the images. For an individual neuron, calcium signal per frame was calculated as an average of all pixels within its cell body mask. This calculation was repeated for each frame in the time series to generate a single-neuron time course. The fluorescent signal (F) was expressed as the percent change relative to the prestimulus baseline (Δ*F*/*F*). For the calculation of averages across neurons, we recorded single-neuron data at a cortical depth of 150 μm (layer II).

### Tissue processing

In accordance with NIH guidelines for the humane treatment of animals, mice were anesthetized with chloral hydrate and perfused transcardially with 0.9 % saline. Brains were removed and divided sagitally. One hemibrain was post-fixed in phosphate-buffered 4 % paraformaldehyde (PFA) at 4 °C for 48 h and sectioned at 40 μm with a Vibratome 2000, while the other hemibrain was snap frozen and stored at −70 °C for protein analysis. All experiments described were approved by the animal subjects committee at the University of California, San Diego (UCSD), and were performed according to NIH recommendations for animal use.

### Immunoblot analysis

The hemibrains were homogenized in Tris-buffered saline (TBS) and ultracentrifuged as previously described [21]. After determining the protein content of all samples by BCA Protein assay (Thermo Fisher Scientific), homogenates were loaded (20 μg total protein/lane), separated on 4–12 % Bis-Tris gels and electrophoresed in 5 % HEPES running buffer, and blotted onto Immobilon-P 0.45-μm membrane using NuPage transfer buffer. The membranes were blocked in 5 % bovine serum albumin (BSA) in phosphate-buffered saline-tween 20 (PBST) for 1 h. Membranes were incubated overnight at 4 °C with primary antibodies against calcineurin (Abcam, 1:1000, rabbit polyclonal), OPA1 (BD Biosciences, 1:1000, mouse monoclonal), MFN1 (Santa Cruz, 1:500, rabbit polyclonal), and mitochondrial-type heat shock protein (mtHSP)70 (BioMol, 1:500, mouse monoclonal). Following visualization, blots were stripped and probed with a mouse monoclonal antibody against actin (1:2000, mab1501, Millipore), as a loading control. All blots were then washed in PBS, .05 % tween-20, and then incubated with secondary species-specific antibodies (American Qualex, 1:5000 in BSA-PBST) and visualized with enhanced chemiluminescence reagent (ECL, Perkin-Elmer). Images were obtained, and semi-quantitative analysis was performed with the VersaDoc gel imaging system and Quantity One software (Bio-Rad).

### Analysis of neurodegeneration

Briefly, as previously described [21], blind-coded, 40-μm-thick vibratome sections were immunolabeled with the mouse monoclonal antibody against microtubule-associated protein-2 (MAP2, dendritic marker, 1:200, EMD Millipore) or the antibody against synaptophysin (synaptic marker, 1:500, Millipore). After overnight incubation, sections were treated with fluorescein isothiocyanate (FITC)-conjugated secondary antibodies (1:75, Vector) or Tyramide Red, (NEN Life Sciences, Boston, MA) transferred to SuperFrost slides (Fisher Scientific), and mounted under glass coverslips with anti-fading media (Vector Laboratories, Burlingame, CA). All sections were processed under the same standardized conditions. The immunolabeled blind-coded sections were serially imaged with a laser scanning confocal microscope (MRC1024, Bio-Rad) and analyzed with the ImageJ program (NIH), as previously described [43, 47]. For each mouse, a total of three sections were analyzed and for each section, four fields in the frontal cortex were examined. This brain region was selected because both patients with HAND and gp120 mice display considerable pathology, and HIV1 gp120 concentrates in this brain region among others (such as the striatum and white matter). Results were expressed as percent area of the neuropil occupied. Additional sets of sections were immunostained with the mouse monoclonal antibodies against NeuN (neuronal marker, 1:500, EMD Millipore), GFAP (astroglial marker, 1:500, EMD Millipore), Iba-1 (microglial marker, 1:5,000, Wako USA, Richmond, VA), or interleukin (IL)6 (Abcam, Cambridge, MA) and developed with diaminobenzidine (DAB). The GFAP, Iba-1, and IL6 immunostained sections were imaged with a digital Olympus microscope (BX51) and analyzed with the Image-Pro Plus program (Media Cybernetics). The NeuN immunostained sections were analyzed as previously described [48] by the dissector method with the SteroInvestigator system.

### ELISA for IL6

For this assay, mouse brain homogenates (20 mg) were prepared and ran with the mouse ELISA kit from Abcam (ab100713). This assay utilizes an antibody specific for mouse IL-6 coated on a 96-well plate. Standards and samples from the mouse brain homogenates treated with vehicle or FK506 were pipetted into the wells. The wells are washed, and biotinylated anti-mouse IL-6 antibody was added. After washing, samples were treated with HRP-conjugated streptavidin followed by washing, TMB substrate, and stop solution. Samples were analyzed in a plate reader for color intensity at 450 nm.

### Immunocytochemical analysis of mitochondrial markers

Briefly, as previously described [21], free-floating 40-μm-thick vibratome sections of mouse brains were washed with Tris-buffered saline (TBS, pH 7.4), pre-treated in 3 % H_2_O_2_, and blocked with 10 % serum (Vector Laboratories), 3 % bovine serum albumin (Sigma), and 0.2 % gelatin in TBS-Tween (TBS-T). Sections were incubated at 4 °C overnight with primary antibodies against calcineurin (Abcam, 1:1000, rabbit polyclonal), OPA1 (BD Biosciences, 1:1000, mouse monoclonal), MFN1 (Santa Cruz, 1:500, rabbit polyclonal), FKBP12 (Abcam, Cambridge MA, 1:1500), or mtHSP70 (BioMol, 1:500, mouse monoclonal). Sections were then incubated in secondary antibody (1:75, Vector), followed by Avidin D-horseradish peroxidase (HRP, ABC Elite, Vector), and reacted with DAB (0.2 mg/ml) in 50-mM Tris (pH 7.4) with 0.001 % H_2_O_2_. Control experiments consisted of incubation with pre-immune rabbit serum. Immunostained sections were imaged with a digital Olympus microscope, and assessment of levels of optical was performed utilizing the Image-Pro Plus program (Media Cybernetics, Silver Spring, MD).

In addition, double immunolabeling studies were performed, as previously described [21], to determine the size and morphology of mitochondria in neuronal cells. For this purpose, vibratome sections of mouse brains were immunostained with antibodies against TOMM40 (Abcam, 1:1000, rabbit polyclonal; red channel) and antibodies against MAP2 (Millipore, green channel). Sections were then reacted with secondary antibodies tagged with FITC to detect MAP2, and with the Tyramide Red amplification system (Perkin-Elmer) to detect TOMM40, FKBP12, and FKBP51. Sections were mounted on superfrost slides (Fisher) and cover-slipped with media containing DAPI. Sections were imaged with a Zeiss 63X (N.A. 1.4) objective on an Axiovert 35 microscope (Zeiss) with an attached MRC1024 laser scanning confocal microscope system (BioRad, Hercules, CA). Digital images were analyzed with the ImageJ program as previously described [21].

### Statistical analysis

All the analyses were conducted on blind-coded samples. After the results were obtained, the code was broken and data were analyzed with the Prism (GraphPad program, La Jolla CA). For the evaluation of statistical significance, independent datasets were compared using two-way ANOVA followed by the Bonferroni multiple comparisons post hoc analysis. *P* values <0.05 were considered significant. All results were expressed as mean ± SEM. Two-photon data were analyzed in MATLAB if they responded to stimulus in at least 13 of 15 stimulus trials using the classic measure of area under the curve (AUC) [42, 49]. For classical shape analysis, calcium transients were aligned based on maximum peak slope and normalized to the maximum peak height. Two-photon imaging results were expressed as the mean ± SEM.

## Results

### FK506 ameliorates neurodegeneration and inflammation in gp120 tg mice

We have previously shown that gp120 tg mice develop neurodegenerative alterations between 6 and 12 months of age [43], which is characterized by, among others, mitochondrial alterations. For this reason, we first analyzed the effects of FK506 on the levels of neuronal markers including NeuN, MAP2, and synaptophysin. As expected, immunostaining with an antibody against the neuronal marker NeuN showed that compared to the non-tg vehicle control, the gp120 vehicle mice displayed a 35 % neuronal loss in the fronto-temporal cortex (Fig. 1a, b). Treatment with FK506 rescued the loss of neurons in the gp120 tg mice (Fig. 1a, b). Immunolabeling and confocal microscopy with an antibody against the dendritic marker-MAP2 (Fig. 1c) and the synaptic marker synaptophysin (Fig. 1e) showed that compared to the non-tg vehicle control, the gp120 vehicle-treated mice displayed a statistically significant 40 % loss of MAP2 (Fig. 1c, d) and 30 % loss of synaptophysin (Fig. 1e, f) in the fronto-temporal cortex. Treatment with FK506 rescued the loss of MAP2 (Fig. 1c, d) and synaptophysin immunoreactivity (Fig. 1e, f) in the gp120 tg mice.

**Fig. 1:** Effects of FK506 on markers of neurodegeneration in gp120 tg mice. Non-tg and gp120 tg mice were treated with vehicle or FK506 for 4 weeks, and immunostained serial vibratome sections were analyzed by digital bright-field microscopy and confocal microscopy. Representative images are shown from the frontal cortex. **a** Representative bright-field microscopic images and **b** computer-aided ImageJ analysis of sections incubated with an antibody against the neuronal marker NeuN showing decreased immunoreactivity in the neocortex in vehicle-treated gp120 tg mice. In vehicle-treated gp120 tg mice, there was a significant decrease (*p < 0.05, by one-way ANOVA post hoc Dunnett’s), while FK506 treatment ameliorated the neuronal alterations compared to vehicle-treated gp120 tg mice (^#^ *p* < 0.05, by one-way ANOVA post hoc Tukey-Kramer). **c** Immunocytochemical analysis and confocal microscopy of sections labeled with an antibody against the dendritic marker MAP2 (FITC channel). **d** Computer-aided ImageJ analysis of the % area of the neuropil that is MAP2 immunostained. In vehicle-treated gp120 tg mice, there was a significant decrease in MAP2 immunoreactivity. **e** Immunofluorescent microscopy and **f** image analysis of the synaptic marker synaptophysin revealed a statistically significant synaptic loss in vehicle-treated gp120 mice compared to vehicle-treated non-tg mice, and treatment with FK506 rescued the synaptic loss in gp120 mice. *Scale bar* = 20 μm. *p value <0.05 by one-way ANOVA and Dunnett’s post hoc analysis compared to vehicle; *N* = 10; age = 12 months of age

Next, we analyzed the effects of FK506 on the levels of neuro-inflammatory markers including GFAP, Iba-1, and IL6. As shown before, immunostaining with an antibody against the astroglial marker, GFAP, showed that compared to the non-tg vehicle control mouse group, the gp120 vehicle-treated mice displayed a 1.5-fold increase in astrogliosis in the fronto-temporal cortex (Fig. 2a, b). Treatment with FK506 partially reduced the astrogliosis in the gp120 tg mice (Fig. 2a, b). Immunolabeling with antibodies against a microglial marker, Iba-1, (Fig. 2a, c) and a pro-inflammatory cytokine, IL6, (Fig. 2a, c) showed that compared to the non-tg vehicle control, the gp120 tg vehicle-treated mice displayed a onefold increase of microgliosis (Fig. 2c) and 50 % increase in IL6 (Fig. 2a, d) in the fronto-temporal cortex. Cells displaying IL6 immunoreactivity were primarily astroglial based on their morphology. Treatment with FK506 reduced the levels of microgliosis (Fig. 2c) and IL6 (Fig. 2d) in the gp120 tg mice. To further confirm the effects of FK506 in inflammation in the gp120 tg mice, ELISA assay to detect IL6 was performed. This study showed an increase in IL6 in the gp120 tg mice compared to controls and a partial recovery following treatment with FK506 (Fig. 2e).

**Fig. 2:** Immunohistochemical and ELISA analysis of the effects of FK506 on markers of neuro-inflammation in gp120 tg mice. Non-tg and gp120 tg mice were treated with vehicle or FK506 for 4 weeks, and serial vibratome sections were treated by immunohistochemistry (IHC) and analyzed by digital bright-field microscopy. Representative images are shown from the fronto-temporal cortex. **a** Photomicrographs of GFAP-, Iba-1-, and IL6-positive astroglial cells in the fronto-temporal cortex of control and gp120 tg mice. **b** Image analysis of the sections showing increase GFAP in gp120 mice vehicle-treated mice, and treatment of gp120 mice with FK506 significantly decreased astrogliosis compared to vehicle-treated gp120 mice. **c** Image analysis of microglial marker Iba-1 showed that vehicle-treated gp120 mice had a statistically significant fold-increase in microgliosis compared to vehicle-treated non-tg mice. Treatment with FK506 significantly reduced the microgliosis in gp120 mice compared to vehicle-treated gp120 mice. **d** Image analysis of cytokine IL6 indicated a statistically significant increase in IL6-immunoreactivity in vehicle-treated gp120 mice compared to non-tg mice. FK506 significantly reduced IL6 levels in gp120 mice compared to vehicle-treated gp120 mice. **e** ELISA assay analysis of levels of IL6 in non-tg and gp120 tg mice treated with vehicle and FK506 showed a statistically significant increase in vehicle-treated gp120 mice compared to non-tg vehicle-treated mice which FK506 treatment significantly reduced. *Scale bar* = 25 μm. *p value <0.05 by one-way ANOVA and post hoc Dunnett’s compared to vehicle; ^#^ *p* value <0.05 by one-way ANOVA and Tukey-Krammer post hoc test compared to vehicle-treated gp120 mice; *N* = 10; age = 12 months of age

Finally, we investigated by immunocytochemistry the levels of the FK506-binding proteins (FKBP) 12 and FKBP51. FKBP12 is a 12-kDa, ubiquitous abundant protein that binds tightly to intracellular calcium release channels and regulates inflammatory responses [50]. The larger members, FKBP51 and FKBP52, interact with Hsp90 and exhibit chaperone activity that is shown to regulate signaling in the CNS and the immune system [24]. FKBP12 immunoreactivity was observed in pyramidal neurons and in the neuropil (Fig. 3a), compared to vehicle, treatment with FK506 increased the levels of FKBP12 immunoreactivity in the non-tg and gp120 tg groups (Fig. 3a, b). Likewise, FKBP51 immunolabeling was observed in the cell body of pyramidal neurons (Fig. 3c); compared to the vehicle-treated group, FK506 increased the levels of FKBP51 immunostaining in the non-tg and gp120 tg groups (Fig. 3c, d). To confirm that FKBP12 and FKBP51 immunolabeling was in pyramidal neurons, double-labeling studies with MAP2 were performed in non-tg vehicle-treated mice (Fig. 3e). Taken together, these results suggest that FK506 engages FKBP that might modulate inflammatory responses in the CNS.

**Fig. 3:** Immunocytochemical and confocal analysis of the effects on FK506-binding proteins in gp120 tg mice. Non-tg and gp120 tg mice were treated with vehicle or FK506 for 4 weeks and immunostained with antibodies against FKBP12 and 51. Representative images are shown from the fronto-temporal cortex. **a** Photomicrographs and **b** image analysis of FKBP12-positive neurons showing that FK506 treatment increased FKBP12 in the non-tg and gp120 tg mice. **c** Photomicrographs and **d** image analysis of FKBP51-positive neurons showing that FK506 treatment increased FKBP51 in the non-tg and gp120 tg mice. **e** Confocal images showing colocalization of FKBP12 (*red*, *upper panel*) and FKBP51 (*red*, *lower panel*), respectively, with dendritic marker MAP2 (*green*). *Scale bar* in **a** = 10 μm. *Scale bar* in **e** = 10 μm. *p value <0.05 by one-way ANOVA and post hoc Dunnett’s compared to vehicle; ^#^ *p* value <0.05 by one-way ANOVA and Tukey-Krammer post hoc test compared to vehicle-treated gp120 mice; *N* = 10; age = 12 months of age

### FK506 rescues the structural mitochondrial alterations in gp120 tg mice

Given that FK506 was neuroprotective in the gp120 tg mice, gp120 mice display mitochondrial alterations [21], and previous studies have shown that calcineurin, a target of FK506, modulates mitochondria; we next analyzed levels of mitochondrial markers in FK506-treated animals using microscopy and biochemical assays. Consistent with previous observations [21], immunolabeling and confocal microscopy with an antibody against the mitochondrial marker TOMM40 showed that compared to the non-tg vehicle control, the gp120 vehicle-treated mice displayed a 45 % increase in the size of the mitochondria (Fig. 4a arrowheads, b), which appeared irregular and appeared abnormally fused in MAP2-positive neurons in the fronto-temporal cortex (Fig. 2a, detail). In contrast, the mitochondria of gp120 tg mice treated with FK506 were comparable to the non-tg controls (Fig. 4a, b). Analysis of levels of MAP2-immunoreactivity was presented in Fig. 1.

**Fig. 4:** Double immunocytochemistry and analysis of the effects of FK506 on mitochondria morphology in neuronal cells. Non-tg and gp120 tg mice were treated with vehicle or FK506 for 4 weeks and vibratome sections double-immunostained with MAP2 (dendritic marker) and TOMM40 (mitochondrial marker) analyzed by digital florescent microscopy. Representative images are shown from the fronto-temporal cortex. **a** Double immunofluorescent microscopy of MAP 2 (*green*) and TOMM40 (*red*) was performed to determine size and morphology of mitochondria in neuronal cells. *White arrowheads* indicate TOMM40-positive reference mitochondria. The detailed images are higher magnification of the *inset box*. **b** Image analysis of mitochondrial marker TOMM40 (*white arrows*) indicated a statistically significant increase in mitochondrial size in vehicle-treated gp120 mice compared to vehicle-treated non-tg mice. FK506-treated gp120 mice had a statistically significant reduction in TOMM40 mitochondrial marker (*white arrows*) indicating a reduction in mitochondrial size compared to vehicle-treated gp120 mice. *Scale bar* = 10 μm; detailed *scale bar* = 1 μm. *p value <0.05 by one-way ANOVA and post hoc Dunnett’s compared to vehicle; *N* = 10; age = 12 months of age

Immunocytochemistry and bright-field microscopy with an antibody against calcineurin showed that calcineurin-immunoreactivity was localized to the neuronal cell bodies and neuritic process in the non-tg and gp120 tg mice (Fig. 5a, b), and no significant differences were detected between non-tg vehicle control and the gp120 tg mice treated with vehicle or FK506 (Fig. 5a, b). Antibodies against mitochondrial proteins such as OPA1, MFN1, and mtHSP70 displayed a granular pattern (arrowheads) of immunostaining in neuronal cells in the neocortex (Fig. 5a). Compared to the non-tg vehicle control, the gp120 tg vehicle-treated mice displayed a statistically significant 40 % loss of the mitochondrial protein OPA1 (Fig. 5a, c) in the fronto-temporal cortex. Treatment with FK506 rescued the loss of OPA1 in the gp120 tg mice (Fig. 5a, c). Levels of MFN1 showed non-significant decrease in FK506-treated non-tg mice and a trend toward an increase in vehicle-treated gp120 tg mice compared to non-tg mice (Fig. 5a, d); treatment with FK506 led to a statistically significant increase in levels of MFN1 in gp120 tg mice (Fig. 5a, d). Levels of mtHSP70 were comparable among the four groups, and no effects of FK506 were detected (Fig. 5a, e).

**Fig. 5:** Immunocytochemical analysis of the effects of FK506 on the FK506-binding protein, calcineurin, and markers of mitochondrial fusion in non-tg and gp120 tg mice. Non-tg and gp120 tg mice were treated with vehicle or FK506 for 4 weeks, and serial vibratome sections were immunostained and analyzed by digital bright-field microscopy. Representative images are shown from the frontal cortex. Calcineurin is an FK506-binding protein, and OPA1 and MFN1 are GTPases that are required for mitochondrial fusion. *Black arrowheads* indicate the granular staining pattern. **a** Representative bright-field microscopic images and **b** computer-aided ImageJ analysis of sections incubated with antibodies against calcineurin, which was unaffected by mouse type or treatment, while **c** OPA1 was significantly decreased in vehicle-treated gp120 tg mice compared to vehicle-treated non-tg mice. Treatment of gp120 mice with FK506 rescued the loss of OPA1. **d** Levels of MFN1 were significantly increased in FK506-treated gp120 mice compared to vehicle-treated non-tg mice. **e** mtHSP70 was included as a control protein and was unaffected by treatment or mouse type. *Scale bar* = 20 μm. *p < 0.05, by one-way ANOVA post hoc Dunnett’s; ^#^ *p* < 0.05, by one-way ANOVA post hoc Tukey-Kramer. *N* = 10; age = 12 months of age

In order to verify these results by an independent approach, immunoblot analysis was performed with membrane fractions from each of the four genotype/treatment groups. Calcineurin was detected as a single band at approximately 59 kDa (Fig. 6a). Levels of calcineurin were comparable among the four groups, and no effects of FK506 were detected (Fig. 6a, b). OPA1 was detected as a doublet at approximately 90 kDa. Compared to the non-tg vehicle control, the gp120 tg vehicle mice displayed a non-significant 20 % decrease in OPA1 (Fig. 6a, c), and treatment with FK506 significantly increased the OPA1 levels in the gp120 tg mice (Fig. 6a, c). MFN1 was detected as a doublet at approximately 70–80 kDa (Fig. 6a). Levels of MFN1 showed a trend toward an increase in vehicle-treated gp120 tg mice compared to non-tg mice (Fig. 6a, d), and treatment with FK506 significantly increased levels of MFN1 in gp120 tg mice (Fig. 6a, d). mtHSP70 was detected as a single band at approximately 72 kDa (Fig. 6a). Levels of mtHSP70 were comparable among the four groups of mice (Fig. 6a, e).

**Fig. 6:** Immunoblot analysis of the effects of FK506 on the FK506-binding protein, calcineurin, and markers of mitochondrial fusion in non-tg and gp120 tg mice. Non-tg and gp120 tg mice were treated with vehicle or FK506 for 4 weeks and were analyzed by immunoblot. **a** Representative Western blots are shown from the membrane fraction of whole brain lysate that was immunoreacted with antibodies against calcineurin, an FK506-binding protein, OPA1 and MFN1, GTPases that are required for mitochondrial fusion, and mtHSP70, a mitochondrial housekeeping control protein. **b** Computer-aided analysis of sections incubated with an antibody against calcineurin, which was unaffected by mouse type or treatment. **c** OPA1 was detected as a doublet which was non-significantly decreased in vehicle-treated gp120 tg mice compared to vehicle-treated non-tg mice. Treatment of gp120 mice with FK506 led to a statistically significant increase in OPA1 compared to vehicle-treated non-tg mice. **d** Levels of MFN1 were detected as a double tat approximately 70–80 kDa and were significantly increased in FK506-treated gp120 mice compared to vehicle-treated non-tg mice. **e** mtHSP70 was detected as a single band, was included as a control protein, and was unaffected by treatment or mouse type. *p < 0.05, by one-way ANOVA post hoc Dunnett’s; ^#^ *p* < 0.05, by one-way ANOVA post hoc Tukey-Kramer. *N* = 10; age = 12 months of age

### FK506 ameliorates the hyperactivity in gp120 tg mice but no effects of calcium imaging by two-photon microscopy

Next, we investigated the functional effects of FK506 in the gp120 tg mice both in the open field and by calcium live imaging. As previously described [51], we found that compared to non-tg vehicle, the gp120 tg vehicle-treated mice were hyperactive in the open field as reflected by the increase beam breaks (Fig. 7a) and distance traveled (Fig. 7b); treatment with FK506 recovered the levels of activity back to the baseline (Fig. 7a, b). However, levels of thigmotaxis (time expended in borders of the cage vs. the center) and rearing were comparable among the four groups of mice, and no effects of FK506 were detected (Fig. 7c, d).

**Fig. 7:** Effects of FK506 treatment on behavior in non-tg and gp120 tg mice. Four behaviors were evaluated in the open field test: total activity, total distance, thigmotaxis, and rearing. **a** Vehicle-treated gp120 tg mice were hyperactive compared to non-tg mice, and FK506 treatment significantly reduced the activity levels compared to vehicle-treated gp120 tg mice. **b** Vehicle-treated gp120 tg mice covered a significantly greater total distance compared to vehicle-treated non-tg mice. **c** Thigmotaxis and **d** rearing were not significantly different between mouse type or treatment group. *Scale bar* = 10 μm. *p < 0.05, by one-way ANOVA post hoc Dunnett’s. *N* = 10; age = 12 months of age

Since we have previously shown that in various models of neurodegeneration the mitochondrial calcium buffering capacity is abnormal and this is recovered by FK506 [42], next we investigated if the gp120 tg mice displayed similar deficits and if FK506 will rescue the defects. For this purpose, the barrel cortices of non-tg and gp120 tg mice were analyzed using the 1-Hz stimulus paradigm and a depth of 150 μm (Fig. 8). Neurons, labeled with calcium indicator Oregon green 488 BAPTA (OGB1), appeared in green (Fig. 8a). Astrocytes, labeled with both OGB and SR101, appeared in yellow (Fig. 7a), or as white (Fig. 8b). The masks for the region of interests (ROIs) for neurons and astrocytes (Fig. 8c) were used for the initial processing of individual calcium traces (Fig. 8d). Calcium transients were normalized for peak shape in order to evaluate the peak shapes using AUC. Under the 1-Hz stimulus paradigm and at a depth of 150 μm, the calcium transients from the gp120 tg mice with and without FK506 treatment had geometric shapes indistinguishable from the non-tg mice (Fig. 8e). Similarly, the AUCs were indistinguishable from non-tg mice (Fig. 8f). Taken together, these results suggest that independent of calcium currents, FK506 rescues the neurodegenerative, mitochondrial pathology, and hyperactivity behavior in the gp120 tg mice.

**Fig. 8:** Calcium dynamics by live imaging in the barrel cortex neurons in gp120 tg mice treated with FK506. **a** Composite two-photon image of the calcium indicator dye, OGB (*green*), and astrocyte marker, SR101 (*yellow-orange*). Representative two-photon images indicating the SR101-positive structures in each mouse type. Regions of interest for each image were extracted; neurons are indicated in *green* and astrocytes are in *red*. **b** The time course for the calcium signal was extracted based on regions of interest identified in the previous panel for 1 Hz. The *arrows* indicate the onset of the stimulus. **c** Visual representation of average calcium peak shapes for non-tg, GP120, and GP120 mice treated with FK506 mice using 1Hz stimulus frequency at a depth of 150 μm. **d** There was no significant difference between normalized calcium traces from barrel cortex neurons that were quantified using area under the curve (AUC). *Scale bar* for photomicrographs is 10 μm

## Discussion

Immunophilin ligands such as cyclosporine A, rapamycin, and FK506 are well-known immunosuppressive drugs widely used in transplantation medicine. These compounds have also been utilized or investigated as treatments for various types of cancer, hepatitis C, and as neuroprotective agents [52]. We have recently shown that FK506 rescues the mitochondrial calcium buffering defects in PD α-synuclein models [42], and for the present study, we investigated the neuroprotective properties of FK506 in a model of HIV-1 gp120-mediated neurotoxicity. Here, we show that FK506 reduced the neuronal damage and neuro-inflammation in the gp120 tg mice. Moreover, while vehicle-treated gp120 tg mice displayed damaged mitochondria and increased markers of neuroinflammation, FK506 rescued the morphological mitochondrial alterations, decreased levels of GFAP and Iba1, and increased FKBP12 and 51.

These results are consistent with previous studies showing that FK506 is neuroprotective in models of stroke [53], spinal cord injury [54], and neurodegeneration [41], including models of PD [55, 56], AD [24], and HD [25]. FK506 has also been found to be protective in a model of antiretroviral toxic neuropathy [57]. Several mechanisms of action have been proposed to explain the neuroprotective effects of FK506 [35]. For example, it has been shown that FK506 effects might be mediated by a large family of co-chaperone proteins called the FK506-binding proteins (FKBPs) [35]. Recently, changes in the levels of FKBP51 and FKBP52 have been correlated with short-term recognition memory impairment in aged mice [58]. Since all FKBPs including FKBP51 and FKBP52 contain a domain with prolyl cis/trans isomerase (PPIase) activity [24], when FK506 binds to this domain, it inhibits their PPIase activity and prevents mitochondria from calcium overload while also modulating immune suppression by blocking calcineurin. Along these lines, in the present study, we found that FK506 increased levels of FKBP12 and 51 in the non-tg and gp120 tg mice, proteins involved in the anti-inflammatory and neuro-modulatory effects of FK506.

Another neuroprotective mechanism that has been proposed for FK506 involves the FKBPs interact with Hsp90 and exhibit chaperone activity that might be responsible for the neuroprotective effects [24]. Protein dephosphorylation by calcineurin plays an important role in neuronal signaling relevant to the regulation of calcium channels, glutamate release, and synaptic plasticity. In vitro, FK506 protects cortical neurons from NMDA-induced death and promotes phosphorylation of nitric oxide synthase thereby inhibiting its activity and nitric oxide synthesis. FK506 also inhibits p38 MAPK-mediated inflammation [39, 40]. However, it is less clear if this mechanism is as relevant in vivo, and the potential anti-inflammatory effects of FK506 have been proposed as a potential neuroprotection mechanism [59]. For the present study, we showed that in addition to protecting the neuronal architecture from gp120 neurotoxicity, FK506 reduced inflammation as assessed by immunostaining with antibodies against GFAP, Iba1, and IL6. Our findings are in agreement with previous studies, which have shown that FK506 targets astrocytes and microglia and modulates neuro-inflammation ischemia and neurodegeneration [53]. FK506 reduced IL-1β, IL-6, and TNF-α expression in models of stroke and inhibited the lipopolysaccharide-induced activation and cytokine expression in microglia in vitro [53].

Another FK506-induced mechanism involves the activation of autophagolysosomal pathways that enhance the clearance of aggregated misfolded proteins such as PrPsc [60]. In this study, FK506 increased the levels of autophagy-related molecules such as LC3-II, ATG12-ATG5, and ATG7. In the gp120 tg mice, we have previously shown alterations in autophagy [61]; however, the effects of FK506 in this pathway in gp120 tg mice are unclear; future studies will address this question. Furthermore, recent studies have suggested that FK506 acts at the level of the mitochondria by modulating abnormal cytosolic and mitochondrial Ca^2+^ dynamics [37]. FK506 has also been shown to decrease the ionophore-induced rise in [Ca2+]i in both neurons and astrocytes [62]. Along these lines, it has been shown that FK506 reduces mitochondrial-dependent apoptotic cell death induced by 3-nitropropionic acid in neuronal cultures [63]. Likewise, we have recently reported that FK506 rescues the alterations in the mitochondrial-dependent calcium buffering capacity in amyloid precursor protein, α-synuclein, and microtubule-associated protein tau tg mice [42]. For the present study, we found that neuroprotective effects of FK506 were associated with the amelioration of the mitochondrial morphological and biochemical alterations in the gp120 tg mice. Moreover, we found improvements in the hyperactivity in the gp120 tg mice. However, while previous in vitro studies indicate that gp120 triggers calcium alterations [14], by two-photon microscopy, there were no apparent abnormalities in calcium transients in gp120 tg mice. The current findings are, however, consistent with previous studies [21], in which we found that in HAND and gp120 tg mouse model levels of MFN1 are increased. MFN1 is a dynamin-related protein of the outer mitochondrial membrane that functions in concert with OPA1 to regulate mitochondrial fusion [64], a function that cells may utilize to dilute the contents of damaged mitochondria in response to stress and prevent apoptosis [65]. In the current study, FK506 further enhanced MFN1 expression. This suggests that the beneficial effects of FK506 in this model of HIV1 neurotoxicity might be independent of calcium and be more closely related to the regulation of neuroinflammation and mitochondria. Future analyses will focus more closely on the anti-inflammatory and autophagy-modulating mechanisms of FK506. As in the general fight against HIV infection, and in this study, therapies that target multiple cellular processes may be the most effective at treating HIV-induced neurodegeneration.

## Conclusions

We found that FK506 is neuroprotective in the gp120 tg model most likely by reducing inflammation and improving mitochondrial morphology. Together, these results suggest that FK506 might be potentially useful in the therapeutic management of patients with HAND.

## Abbreviations

AD, Alzheimer’s disease; AUC, area under the curve; BSA, bovine serum albumin; cART, combined antiretroviral therapies; DAB, diaminobenzidine; DRP, GTPase dynamin-related protein; F, fluorescent signal; FITC, fluorescein isothiocyanate; FK506BP, FK506-binding proteins; FOV, field of view; GFAP, glial fibrillary acidic protein; HAND, HIV-associated neurocognitive disorders; HD, Huntington’s disease; HIVE, HIV encephalitis; IL, interleukin; IP, intraperitoneal; ISI, interstimulus intervals; MAP2, microtubule-associated protein-2; MAPK, mitogen-activated protein kinase; MFN, mitofusin; mtHSP, mitochondrial-type heat shock protein; OGB, Oregon green 488 BAPTA; OPA, optic atrophy; PBS, phosphate-buffered saline; PBST, phosphate-buffered saline-tween 20; PD, Parkinson’s disease; PFA, paraformaldehyde; PPlase, prolyl cis/trans isomerase; ROI, region of interest; TBS, Tris-buffered saline; TBST, TBS-Tween; tg, transgenic; UCSD, University of California, San Diego.
